RETRACTED

# Intelligent Recommendations of Startup Projects in Smart Cities and Smart Health Using Social Media Mining

**DOI:** 10.1155/2021/3400943

**Published:** 2021-09-24

**Authors:** Wahiba Ben Abdessalem Karaa, Eman Alkhammash, Thabet Slimani, Myriam Hadjouni

**Affiliations:** ^1^Department of Computer Science, High Institute of Management, University of Tunis, 2000 Bardo, Tunis, Tunisia; ^2^RIADI-GDL Laboratory, ENSI, University of Manouba, 2010 Manouba, Tunisia; ^3^Department of Computer Science, College of Computers and Information Technology, Taif University, P.O. Box 11099, Taif 21944, Saudi Arabia; ^4^Department of Computer Science, College of Computer and Information Science, Princess Nourah Bint Abdulrahman University, P.O.Box 84428, Riyadh, Saudi Arabia

## Abstract

The paper presents a recommendation model for developing new smart city and smart health projects. The objective is to provide recommendations to citizens about smart city and smart health startups to improve entrepreneurship and leadership. These recommendations may lead to the country's advancement and the improvement of national income and reduce unemployment. This work focuses on designing and implementing an approach for processing and analyzing tweets inclosing data related to smart city and smart health startups and providing recommended projects as well as their required skills and competencies. This approach is based on tweets mining through a machine learning method, the Word2Vec algorithm, combined with a recommendation technique conducted via an ontology-based method. This approach allows discovering the relevant startup projects in the context of smart cities and makes links to the needed skills and competencies of users. A system was implemented to validate this approach. The attained performance metrics related to precision, recall, and F-measure are, respectively, 95%, 66%, and 79%, showing that the results are very encouraging.

## 1. Introduction

### 1.1. Background

Sustainability aims to improve life quality without troubling environmental safety [1]. Various studies have shown that smart city projects are always concerned with sustainability objectives [2, 3]. Smartness and sustainability are interrelated in city strategies [4, 5]. Smart city projects, today, give forefront attention to sustainability when producing technological-based services [6]. Many studies have focused on difficulties related to smart sustainable city projects' startup phase, especially for young people in developing countries [7].

Smart city services integrate many greatly promising technologies resembling databases, data warehouses, advanced computer networks, content management, big data, social mining, and so forth [8]. It should be noted that these technological solutions in the field of smart cities have been applied in various areas, such as smart home [9], smart grid [10], smart community [11], smart governance [12], smart building [13], smart manufacturing [14], smart agriculture [15], and smart healthcare applications that play an important role nowadays [16–18]. Smart healthcare monitoring in smart cities is important to provide better services and carefulness to residents [19–23].

RETRACTED

Social media is one of the most recent and rapidly growing phenomena. Social media platforms have become popular in users' daily lives; they allow communication and sharing of opinions and experiences [24]. The data collected from social media are particularly useful and reflect significant human experiences and behaviors for the resolution of various problems. Many researchers have proposed social media mining for data collection in the context of smart city applications, needed as a complement to data collected from sensors to ensure efficient services [25].

Social media can provide help to healthcare, since everybody with access to social media can post information about how to deal with certain health problems [26, 27]. The use of data of Twitter, Instagram, and so forth has been exploited to investigate, track, and predict a range of health incidences and diseases [28–30].

### 1.2. Motivation

The numbers of approaches and applications using social networks, in the context of smart cities, constantly increase to measure resident engagement [31], to guarantee security for citizens and detect violence [32], to manage traffic and emergency services [33], and to do transport planning [34]. Numerous studies and applications have been interested in social media and their impact on smart cities, such as Twitter emotion analysis [35], detection and classification of critical events [36, 37], and education [38, 39].

The collected information from social networks can be mined to understand the links between smart cities' social and technical aspects. Indeed, social media exploitation provides the necessary tools to analyze information diffusion, analyze social behavior vis-à-vis smart cities, study its influence, and provide effective recommendations.

### 1.3. Contribution

In this research work, we focus on the recommendation of startup projects in the context of smart cities for Saudi youth, based on what users have posted in tweets. These tweets can be seen as raw resources and reach information exchanged between individuals. Thus, this work focuses on designing and implementing an approach for processing and analyzing tweets inclosing data related to smart city startups. The objective is to provide recommendations to users about smart city and smart health startups to improve entrepreneurship and leadership following their skills and competencies.

RETRACTED

For this purpose, first, extracted tweets are preprocessed (cleaning, stop word removal, tokenization, and lemmatization). Then, the Word2Vec algorithm is applied; it uses a neural network model to learn word associations from the preprocessed tweets. From the model, synonymous words are detected and represented in a vector based on cosine similarity. The vector indicates the level of semantic similarity between the words. In this study, this vector conveys similar words related to the names of smart city startups.

Finally, from the Word2Vec vector, some recommendations are given to encourage Saudi youth to focus on startup projects related to smart cities to enhance the quality of life for KSA citizens with Vision 2030. In this study, the recommendations are based on an OWL ontology created for this purpose. Besides, for each recommended project, a list of needed skills are suggested to support the user's choice according to his skills and competencies.

### 1.4. Paper Organization

This paper is organized as follows. The second section will deal with a literature review about the KSA's position regarding innovation and smart city startups and recommendation techniques for startup projects after the first introductory section. The subsequent third section is dedicated to a presentation of the research methodology and the proposed approach. After that, the fourth section will discuss the research findings, based on the experimentations and tests and evaluations of the implemented system. The final section, Conclusion, will emphasize some future works to enhance the attained results.

## 2. Literature Review

### 2.1. KSA's Position Regarding Innovation and Smart City Startups

To encourage entrepreneurship and improve the technological innovation of youths in the Kingdom of Saudi Arabia (KSA), many strategies have been formulated, following the social development to join efforts and achieve the goals and programs of Vision 2030. The government constantly promotes innovation partnership programs, allowing ambitious youth entrepreneurs to work on innovative startup projects. With international strategic engagement, the government encourages emerging projects that intersect with sustainable development objectives. The government offers financial support for implementing these projects by providing the necessary assistance and contributions to carry out their projects, especially for young people [40]. This support leads to the country's advancement and the improvement of national income, improving quality of life and reducing unemployment.

RETRACTED

There are many classes of organizations that are specialized in financial funding for small projects in KSA. The first actor is the bank sector [41].

However, even though youth project funding organizations are abundant, and with the large panoply of businesses that exist on the scene and the growth of competitiveness, there are problems associated with choosing the best project or investment. The decisions to be taken may have consequences on the development of the project and its success. Young people generally lack experience; it is hard for them to find suitable startups. Numerous recommendation algorithms can be operated to recommend suitable things to users based on diverse information, such as the context and preferences. A recommendation system can help Saudi youth find a suitable smart city and sustainable startups.

### 2.2. Recommendations for Smart City Service Startups

There are commonly known recommendation algorithms that can be applied or adapted to different fields [42, 43]. The most recommender approaches are as follows: based on Collaborative Filtering (CF) [44, 45] and Content-Based (CB) [46].

The prosperity of a business and the investment returns depend on the startup's choice. Hence, recommender approaches related to startup projects have received increasing consideration. They can be beneficial for youth entrepreneurship and increase the country's economic benefits [47].

The majority of proposed recommendation approaches in the startup field use the CF, the CB, or hybrid methods [48]. To rank the startups and recommend them to investment companies, Xu et al. [49] used collected data about investment companies, startup projects, and investment events. Kim et al. [47] suggested a framework that recommends expected startups to enterprises based on their technological similarity scores between patent abstracts and startup profile texts by collecting patent applications from the WISDOMAIN website and startup information from “Crunchbase” database. Zhong et al. [50] proposed an integrated approach to recommend a startup investment to investors by studying the investor's investment preferences and the expected returns and potential risks of the startup. The proposed approach analyzes investment events collected from the “ITjuzi” platform.

Social network exploration has been employed in many fields with diverse goals. Many researchers have demonstrated that information from social networks can be exploited to improve the accuracy of recommendation systems [51–53]. However, social networks have never been exploited in the recommendation of startup projects. Even so, there is plenty of quantity of exchanged information between users, in social networks, about startup projects, which can be exploited in many domains, particularly, in startup recommendation systems, in the context of smart cities subsections if several methods are described.

RETRACTED

## 3. Materials and Methods

The methodology adopted in this study derives from studies and considerations of smart city sustainable services, social networks, startups, and recommendation systems. The following objectives guide the proposed approach:

- Provide opportunities to young people and encourage them to instigate their startup project in the context of smart cities.
- Establish a startup recommendation system in the context of smart cities to guide young people in their choices.
- Take advantage of the great information about startup projects in social networks to establish such a recommendation system.

This research work focuses on the design and implementation of an approach concerned with processing and analyzing tweets holding data associated with startup projects about smart cities to provide recommendations for the Saudi Youth towards enhanced entrepreneurship and leadership.

The proposed approach sets up an association between different research fields and suggests a recommendation system for smart city startups by mining tweets about smart cities. The proposed approach uses a Twitter mining approach and ontology-based recommendation technique to extract information from tweets, gives recommendations, and provides useful information to Saudi youth, connecting them to smart city growth and engaging them in innovation projects.  Figure 1 illustrates the main components of the proposed approach.

The proposed approach baptized “RecSPSC” entails four main components: tweets extraction, tweets preprocessing, tweets representation, and recommendation module. The first component performs the collection of public tweets through an application programming interface (API). In the second module, the collected tweets are preprocessed and passed to the tweets representation module. In this third module, data is fed into a neural network (Word2Vec) to discover a potential correlation between the different encountered concepts. The output is a vector of words representing the semantic similarity between these words.

Finally, the previous step's output is used as an input in the fourth module to make recommendations based on a startup-ontology. The ontology represents the concepts related to innovation and smart city service startups and skills associated with these projects. The following subsections reveal the details of each component of the proposed approach RecSPSC.

RETRACTED

### 3.1. Extraction of Tweets

According to statistics [54, 55], as of April 2020, Twitter, the online social networking, was ranked as one of the most important social networks, based on active users. As of this date, Twitter had 386 million active users. Tweets are short messages spread between twitter platform users. An author's tweets are dispersed to his followers or subscribers, that is, individuals who have chosen to follow his messages' publication. We introduce the following example:

RT @BlueprintStats receives $20K from the Community Ideation Fund in the Velocities region. Read more about the sports technology #startup, CEO @hunterhawley5, and the company's plans looking forward.

The Twitter messages have a maximum of 280 characters including the following:

- Text or the message, in a given language, to transmit.
- A Hashtag, the symbol #, followed by a set of relevant words or characters. The hashtags usually boost the audience of a tweet and help Twitter users in searching for tweets.
- The username such as @username: to indicate the author of the tweet.
- Image or video. These types of multimedia tweets are habitually well spread.
- Optionally, a URL related to an interesting link, providing more details about the subject since the tweet length is limited. The addition of a link can also increase the audience of a tweet.

Apart from the general tweets, we can find mentions, replies, and retweets, which are tweets but with particularities: the mention is a tweet containing the username of another Twitter account preceded by the @ symbol. For example, “Hello @TwitterSupport!.” The reply is a reaction to another person's tweet. Mentions and replies are displayed to the recipient in their notifications tabs. Only people who follow the sender and follow the mentioned account will see these tweets in their home timeline (the timeline is the main page that shows the tweets of accounts to which the user has subscribed). For the sender, they will be displayed on their profile page containing their public tweets.

A retweet is a reposting of a tweet. Retweets help to share tweets with followers. Anyone can retweet someone else's tweets or his tweets. The users type “RT” at the commencement of a tweet to indicate that they are retweeting someone else's tweet.

In practice, Twitter has its specific vocabulary; Twitter users create many hashtags in abbreviations. The most commonly used are identified as follows:

#TT, Trending Topics; #FF, FollowFriday (every Friday, Twitter accounts that you wish to recommend to subscribers of your feed); #PP, Profile Picture; #NP, Now Playing (used to talk about the music we are listening to (music, radio…)); #NW, Now Watching (used to talk about what we are watching: television, film, videos…); #LT, Last Tweet (or the previous tweet, used when a user refers to his previous posted tweet); #NSFW, Not Safe For Work (used to report inappropriate content in a professional or public setting, indecent, even vulgar, violent, or sexual).

RETRACTED

In addition to the text message itself, a tweet can have more than 150 hidden attributes related to it, including a unique identifier for the tweet, the time when this tweet was created, the geographic location of the tweet, the number of times the tweet has been replied to, and the number of times the tweet has been retweeted.

For the collection of tweets, we used TAGS (Twitter Arching Google Spreadsheet) to fetch Twitter data related to three months (from 16 June 2020 to 16 June 2021), with hashtags in English, such as #smart city, #Sustainability, #investor, #startup, and #entrepreneur, and Arabic, such as (Pilot project) مشروع ريادي#, (Support projects) دعم مشاريع#, (Investor) مستثمر#, (Initiative) مبادر#, and (startup) شركات ناشئة #. We also search tweets using terms without #, such as smart city, support project, investor, and ناشئة. We collected in an excel sheet 1 529 775 nonduplicated tweets (Table 1).

Although the words and hashtags used to collect the tweets were in English and Arabic, we got tweets in other languages, such as French, Italian, and Japanese. In Table 2, a sample of extracted tweets with the hashtag “startup” are given.

### 3.2. Preprocessing of Tweets

As explained in Algorithm 1, the preprocessing tasks on the extracted tweets are translation, cleaning, tokenization, and lemmatization.

#### 3.2.1. Translation

Although the aforementioned hashtags and terms used to collect the tweets were in English and Arabic, we got tweets in many other languages. For this reason, a translation of the tweets to English is required.

#### 3.2.2. Cleaning the Tweets

As explained in the previous section, apart from the tweet's text, many other elements are found, such as username, image, video, URL, mention, reply, retweet, and abbreviations. These elements are not relevant in this study and need to be removed. The tweet cleaning consists of the following steps:

- Remove the abbreviations, such as #TT, #FF, and #PP, as well as the abbreviation “RT” referring to retweets.
- Remove extra whitespaces (when there is more than one space between words).
- Remove usernames, which are portions of text starting the symbol “@” without spaces in the middle.
- Remove URLs, which are links to websites. These links are considered portions of text with www, http://, or https:// in the beginning, without spaces in the middle.
- Remove numbers.
- Remove punctuation.
- Remove hashtags and nonalphabet characters (?,؟ $, {, ŭ, ȸ, etc.).
- Transform the tweets into lower cases.
- Remove the stop-words (a, and, or, etc.).

RETRACTED

#### 3.2.3. Tokenization

It is an essential step in natural language processing. It identifies the basic units (words) to be processed in a given language [56]. Generally, tokenization is based on the presence of special delimiters or marks, such as spaces.

#### 3.2.4. Lemmatization

It is the process of converting a word into a normalized form. It consists of removing the suffix of a word [57, 58]. For instance, by removing the words' suffixes, ranked, and ranks, we get the lemma rank. This step is very useful for many natural languages' processing to reduce the size of the vocabulary.  Table 3 shows samples of tweets after the stated steps of the preprocessing module.

### 3.3. Vector Representation

Word2vec [59, 60] is a neural network with an input layer, one hidden layer, and an output layer. It is an unsupervised machine learning method that automatically learns from the neighboring words (context) in the input corpus and represents words into vectors, according to their similarities. Word2Vec [61, 62] takes a text corpus as input and produces a vector with semantic and syntactic similarities for each word in the corpus. For each word in the corpus, a vector is represented grouping the words that are sharing the same context (Figure 2).

Word2vec [47, 50] can be implemented according to two approaches, the Continuous Bag-of-Words Approach (CBOW) or the Continuous Skip-Gram Approach (Skip-Gram) [63]. The CBOW uses the context to expect a target word. For example, it predicts the output word from other near words. Skip-Gram uses a word to guess a target context, for example, predicting other words that appear around a given word (Figure 3).

The two approaches need a large corpus to capture relationships between words in their contexts and have the same neural network architecture and the same parameters. Generally, CBOW is used when the corpus is too large; it does faster and better than Skip-Gram in this situation.

In this paper, a CBOW-based approach is used. In CBOW, the iterative training process tends to maximize the log probability of each word given its context using the following equation [59, 60]:

(1) $$\begin{array}{c} \max\frac{1}{T}\;\sum_{t=1}^{T}\log\;p\left(wt|w_{t-c}^{t+c}\right), \end{array}$$

where *T* is the corpus size; *wt* is the *t*^th^ word in the corpus; *c* is the window size; it is a given number of words surrounding the input word. *w*_*t*−*c*_^*t*+*c*^ is the set of words in the window of size *c* surrounding *wt*, where *p*(*w*_*t*−*c*_^*t*+*c*^) is a softmax function, computed as follows:

(2) $$\begin{array}{c} p\;\left(wt_{t-c}^{t+c}\right)=\frac{\exp\left(e_{wt}^{\prime T}\right).\sum_{-c\leq j\leq c,j\#0}e_{wt+j}}{\sum_{w}\text{exp}\left(e_{wt}^{\prime T}\right).\sum_{-c\leq j\leq c,j\#0}e_{wt+j}}, \end{array}$$

where *ew* and *e*′*w* signify, respectively, the input and output embeddings in CBOW.

RETRACTED

Since tweets are collected using specific hashtags and terms (smart city, startup, sustainability, etc.), these words tend to appear together in the tweets, and the sought names of startup projects will have similar contexts. Word2Vec asserts that words sharing similar contexts share semantic meanings as well. Consequently, we can state that Word2vec using the CBOW approach can be useful to embody the tweets' frequent words and represent their relationships. The relationships are computed giving the similarity. The similarity of two words is computed according to the cosine similarity of two vectors that represent the two words. Consider vectors v1 and v2, related to two given words. The cosine similarity between the words is obtained by taking the scalar product of the two vectors divided by the product of their norms (equation (3)).

The value of a cosine similarity is included in the interval [−1.1]. The value of −1 indicates opposite vectors, the value of 0 indicates independent (orthogonal) vectors, and the value of 1 indicates colinear vectors with a positive coefficient. The intermediate values are used to assess the degree of similarity.

(3) $$\begin{array}{c} \text{cosine}\left(v1,v2\right)=\;\frac{v1.v2}{\left|\left|v1\right|\right|\;\left\|v2\right\|}. \end{array}$$

In this study, the preprocessed unlabelled tweets are used as a corpus during the training process. All the words are trained alongside other words close to them in the corpus to create a training model. Afterward, in the prediction process, the training model is used to calculate the words' distribution in the corpus. The output is a vector where each element has a distribution of weight towards the other elements. The pseudocode of this step is sketched in Algorithm 2.

The algorithm represents words into vectors based on several features such as vector size, word frequency, windows size, and the number of epochs (Algorithm 2, lines 22 to 25):

- vector_size: This parameter determines the number of neurons in the hidden layer of the network. With vector_size = 2, it will be possible to represent the terms in the plan. We can indicate much more (hundreds of…).
- min_word_frequency: This parameter indicates the minimum frequency of a term included in the calculation to get the most frequent words in the corpus (vocabulary size).
- window_size: This parameter specifies the size of the neighborhood to be taken into account. It fixes the context or a given number of words surrounding the input word in the CBOW model. In the Skip-Gram model, they are the words surrounding the output word.
- epochs: The number of iterations.

RETRACTED

### 3.4. Recommendations of Smart City and Sustainable Startups

Unlike the habitual recommender systems, which generally propose recommender systems to catch useful information such as similar users' preferences on the social network that could be considered by the recommender systems, in this study, the recommender system is based on an OWL ontology. The latter allows the correlation between the different encountered concepts in the tweets and then gives suitable recommendations about smart cities and sustainable startup projects for Saudi youth. The proposed approach RecSPSC is based on the Word2Vec vector from the previous module and a startup-ontology created for this purpose.

Ontologies can be considered valuable tools for the Semantic Web data representation to organize knowledge and explore relationships. In the context of smart cities, ontologies have been used. There have been existing domain ontologies closely related to smart cities and cross-domain ontologies that can help this field. For example, the FIPA (Foundation for Intelligent Physical Agents) device ontology specification is among the early ontologies dealing with devices [64], and OWL-Time [65] is an ontology providing a trivial model for the formalization of temporal objects. The SSN ontology can express sensors regarding measurement processes, capabilities, deployments, and observations [66]. The Stream Annotation Ontology (SAO) [67], as an extension of the SSN ontology, allows the publication of the derived data concerning IoT streams, as well as its capacity to represent aggregated data.

In this work, a new ontology is proposed, which is the startup-ontology. The ontology represents the concepts related to innovation and smart city and sustainable startups as well as future young entrepreneur skills.  Figure 4 defines the concepts of the proposed ontology. The created startup-ontology can be represented with different Syntaxes (OWL/XML, RDF/XML, Turtle, OWL Functional, Manchester OWL, OBO. Latex, and JSON-LD). The url of this ontology is as follows:

 
http://cor.esipfed.org/ont?iri=http://www.startup.com//ontologies/startup.owl

In this study, the effort is concentrated on social media exploitation, which is text tweets. The recommendation technique is conducted through an ontology-based method combined with the Word2Vec algorithm, which can help to discover the relevant concepts related to startup projects in the context of smart cities. It also specifies for the recommended projects the needed skills (Algorithm 3).

RETRACTED

## 4. Results and Discussion

To validate the proposed RecSPSC approach, a system was implemented using Python v3.6 under the PyCharm Integrated Development Environment (IDE). In the first algorithm (Algorithm 1), the preprocessing step includes the following: translation, cleaning of tweets, tokenization, and lemmatization. The Google API was used for the translation of the tweets. The remaining tasks, such as cleaning, as well as tokenization and lemmatization, were carried out with the support of the Natural Language Toolkit (NLTK) libraries [68].

The second algorithm (Algorithm 2) is interested in the generation of the Word2Vec vector. Word2vec algorithm is implemented according to CBOW because of the large number of tweets. The CBOW is implemented with the H2O library. H2O (https://www.h2o.ai/products/h2o/) is a JAVA platform that implements several machine learning algorithms. We can access these functionalities via the API mechanism, in particular under Python.

The third algorithm (Algorithm 3) is related to the recommendation of smart city and sustainable startups that Saudi youth can choose according to the needed skills and competencies for each project. This module required, first, the construction of the ontology and its population. The ontology was created using Protégé, the well-known, free, and open-source framework for building ontologies. The implementation of the recommendation task necessitated the OWLREADY2 library for manipulating the ontology.

The experiments were accomplished by changing the parameters settings of word2vec: vector_size, min_word_frequency, window_size, and epochs.

To evaluate the approach RecSPSC, the experiments are conducted with 1 529 775 collected tweets as mentioned in Section 5.1. Setting vector_size = 2, min_word_frequency = 3, window_size = 1, and epochs = 1000 as parameters, Word2Vec vector is generated.  Table 4 presents an extract of the resulting Word2Vec vector.

For each word in the table, V1 and V2 represent the similarity measure of the word with “startup” in double dimension (vector_size = 2).

We notice that many composed words are concatenated, such as digitalmarketing and artificialintelligence. In the tweets, those words are usually mentioned in the following form: #digitalmarketing and #artificialintelligence. The result can be represented graphically; Figure 5 plots the similarity between the data.

Additional experimentations were performed, varying the parameters (vector_size, min_word_frequency, window_size, and epochs).  Table 5 specifies the size of the generated vectors (Word2Vec size). It is noticed that the Word2Vec size is influenced by the minimum frequency more than by the vector size, the window size, or the number of epochs. For example, with 2, 3, 1, and 1000, respectively, as the vector_size, min_word_frequency, window_size, and epochs, the Word2Vec size is 3065876 (number of words). By changing only the dimension (vector_ size) from 3 to 5, the Word2Vec size is reduced to 28278.

RETRACTED

The generated Word2Vec vector will be used in the recommendation process. The recommender module has as an input the generated Word2vec vector. Indeed, the recommendations vary according to the sated parameters: vector size, the minimum frequency of the words, the window size, and the number of epochs. In Figure 6, the word cloud data visualization is used for representing the recommended smart city service startups. It can be perceived that the most recommended projects are related to marketing strategy, driverless cars, renewables, lifestyle, and so forth.

In addition, for each recommended project, a list of needed skills are suggested to support the user's choice according to his skills and competencies.  Table 6 gathers an extraction of the recommended projects as well as the required skills.

To evaluate and assess the proposed approach's performance, the performance measures, precision, recall, and F-measure, are computed. The precision evaluates the correct smart city service startups recommended by the system from all of those recommended by the system. It measures the aptitude of the system to find only relevant smart city service startups (SCS). It is calculated according to the following equation:

(4) $$\begin{array}{c} \mathrm{precision}=\;\frac{\;c\text{orrect recommended SCS}}{\text{total recommended SCS}}. \end{array}$$

The recall evaluates the total recommended smart city service startups (SCS) from all those available in the corpus (collection of tweets). It is computed according to the following equation:

(5) $$\begin{array}{c} \mathrm{Recall}=\;\frac{\text{total recommended SCS}}{\text{total SCS in the corpus}}. \end{array}$$

The F-measure is synthesizing the precision and recall measures,. It is calculated according to the following equation:

(6) $$\begin{array}{c} F-\text{measure}=\;2*\frac{\text{precision}*\text{recall}}{\text{precision}+\text{recall}}. \end{array}$$

Table 7 summarizes the results of the mentioned performance measures. In line 2, only the minimum frequency is changed. In line 3, the epoch number is modified. In line 4, line 5, and line 6, the window size, vector size, and minimum frequency are changed.

RETRACTED

In Table 7, we can notice that the performances (precision, recall, and F-measure) are influenced by the word frequency taken as a minimum. The lower the frequency, the better the performance. The algorithm performs significantly better when the word frequency is low. We attained the best precision of 0.95, recall of 0.66, and F-measure of 0.79 with three words' frequency, for example. This can be justified by the size of the generated Word2Vec vector, which is larger in the case of low word frequency, and the system generates plentiful potential smart city service startups to feed the ontology-recommender module. We can perceive also that precision is better than recall. This is natural, since there is a correlation between precision and recall; the precision is increased at the cost of the recall. Actually, the system did not detect lots of smart city service startups existing in the corpus. Indeed, many words can be effective smart city service startups but not detected by the system, since they have a frequency less than 3 in the corpus. Commonly, the frequency parameter is chosen to start from 3. With a frequency of 1 or 2, the system will generate a vector of enormous size, where several words are taken into account without being relevant, and therefore the precision will be reduced.

Moreover, Table 7 shows that when the frequency is fixed, five for example, even if we change the other parameters (window size or vector size), the system gives the same size of the generated vector and the same list of words. We can argue that the minimum frequency of words is the most influencing parameter in the generation of the Word2Vec vector.

We evaluated and compared our approach RecSPSC with the widely deployed recommendation approaches, Collaborative Filtering (CF) [44, 45] and Content-Based (CB) [46]. The comparison is performed according to the precision, recall, and F-measure averages (see Table 8 and Figure 7). The results show that RecSPSC outperforms the existing approaches.

## 5. Conclusions

Startups are representatives of innovation as well as new business opportunities. Therefore, great attention is paid to startups in smart cities, since they contribute to the deployment of new products, new services, new business, and so forth and successively lead to the improvement of the life quality and a country's overall economy. This study suggests a novel computational approach for smart city startups' recommendation by identifying the innovation projects from the smart cities' perspectives.

In this approach, tweets are preprocessed. Afterward, the Word2Vec algorithm is applied; it uses a neural network model to learn word associations from the preprocessed tweets. From this model, synonymous words are detected and represented in a vector, based on the cosine similarity. The vector indicates the level of semantic similarity between the words. In this study, this vector conveys similar words related to the names of smart city startups.

RETRACTED

Finally, from the Word2Vec vector, some recommendations are produced to encourage users to focus on startup projects related to smart cities. In this study, the recommendations are based on an OWL ontology created for this purpose. Besides, for each recommended project, a list of needed skills and competencies are suggested to support the user's choice.

The attained performance metrics related to precision, recall, and F-measure are, respectively, 95%, 66%, and 79%, showing that the results are very encouraging. The forthcoming research will focus on further enhancements of the proposed approach. The first main direction for future improvement is related to the Word2Vec algorithm. Actually, the Word2Vec algorithm works with tokens (single word) and generates vectors of tokens with similar characteristics. However, a group of words, called usually “phrase,” carry a special meaning. For instance, “innovation projects,” “support projects,” “digital marketing,” “machine learning,” and “web development” can be relevant in this research as smart city startup projects. The upcoming work will focus on a method that pays special attention to text segmentation to detect sentence boundaries and phrase boundaries (text chunking) and then propose a new algorithm, a Phrase2Vec version, and evaluate its influence on the approach.

In this research, the ontology population is limited. The automatic or semiautomatic ontology population is the second potential work, since the richness of the ontology through its instances can influence the results.

## Figures and Tables

**Figure 1:** The overall approach architecture.

**Figure 2:** Word2Vec representation with 2-dimensional vector.

**Figure 3:** Word2Vec CBOW and Skip-Gram models [53].

**Figure 4:** The proposed startup-ontology.

**Figure 5:** Word2Vec graphical representation.

**Figure 6:** Word cloud representation of the recommended smart city service startups.

**Figure 7:** Comparative curves of performance measures.

**Algorithm 1:** Pseudocode of tweets preprocessing.

**Algorithm 2:** Pseudocode of the generation of words vectors using Word2Vec.

**Algorithm 3:** Pseudocode of the recommendation approach.

**Table 1:** Characteristics of the dataset.

Hashtag and terms	Smart city	Sustainability	Investor	Startup	Entrepreneur	مشروع ريادي	دعم مشاريع	مستثمر	مبادر	شركات ناشئة
Number of tweets	184 564	13 944	877 258	299 803	102 560	23 558	849	13 564	6 465	7 210
Total tweets	1 529 775								

RETRACTED

**Table 2:** Sample of extracted tweets with the hashtag “startup.”

Tweet	Language
How to Replicate Competitor's Backlink strategy? https://t.co/mllmCw0Yoh #socialmedia #digitalmarketing #contentmarketing #growthhacking #startup #SEO #ecommerce #marketing #influencermarketing #blogging #infographic #deeplearning #ai #machinelearning #bigdata #datascience https://t.co/Bdb4DoKvLH	English
On n'a pas la science infuse mais voici nos recommandations ! #Ecologie #Ecoresponsable #Entreprise #Startup https://t.co/39kItrUurL	French
Studierende erhalten jegliche Vorteile &amp; Unterstützung zu Lasten der #Steuerzahler. Wieso erhalten Nichtstudierende nicht dieselben Unterstützungen? #startup #Diskriminierung	German
“ なぜテスラは世界一になった？ トヨタを凌ぐ時価総額 そのカラクリとは(くるまのニュース) - Yahoo!ニュース” #ElonMusk #Tesla #SpaceX #Startup https://t.co/O1ufeG861o	Japanese
RT @victoruxui: Si la situación lo requiere, hacer uso de cards en orden horizontal puede ser mucho más practico que un scroll vertical con…	Spanish
Ci vediamo martedì 7 luglio alle ore 18:30 all'evento online, organizzato da @founding, dove proveremo a der il nostro piccolo supporto alle #startup in phase di pre-seed partecipanti al programma di accelerazione. Per partecipare l'iscrizione è gratuita	Italian
انا عن نفسي، اكتشفت قوتي في المشاريع التقليدية، التقليدية اقصد فيها انه ماهو مشروع ريادي جديد يحل مشكله جديدة، مافي مشروع قد سبقة فيها. وجدا ما اطيق ولا احب ادخل مشروع ريادي جديد ما فيه منافسين!	Arabic

**Table 3:** Examples of preprocessed tweets.

Original tweets	Preprocessed tweets
How to Replicate Competitor's Backlink strategy? https://t.co/mllmCw0Yoh #socialmedia #digitalmarketing #contentmarketing #growthhacking #startup #SEO #ecommerce #marketing #influencermarketing #blogging #infographic #deeplearning #ai #machinelearning #bigdata #datascience https://t.co/Bdb4DoKvLH	replicate competitor backlink strategy socialmedia digitalmarketing contentmarketing growthhacking startup ecommerce market influencermarketing blogging infographic deeplearning machinelearning bigdata datascience
On n'a pas la science infuse mais voici nos recommandations ! #Ecologie #Ecoresponsable #Entreprise #Startup https://t.co/39kItrUurL	dont infuse science recommendations ecology ecoresponsible company startup
Studierende erhalten jegliche Vorteile &amp; Unterstützung zu Lasten der #Steuerzahler. Wieso erhalten Nichtstudierende nicht dieselben Unterstützungen? #startup #Diskriminierung	studierende erhalten jegliche vorteile unterst tng lasten steuerzahler wieso erhalten nichtstudierende nicht dieselben unterst tngen startup diskriminierung
“ なぜテスラは世界一になった？ トヨタを凌ぐ時価総額 そのカラクリとは(くるまのニュース) - Yahoo!ニュース” #ElonMusk #Tesla #SpaceX #Startup https://t.co/O1ufeG861o	tesla become world market capitalization surpass toyota karuma newsyahoo news elonmusk tesla spacex startup
RT @victoruxui: Si la situación lo requiere, hacer uso de cards en orden horizontal puede ser mucho más practico que un scroll vertical con…	situation require use card horizontal order much practical vertical scroll
Ci vediamo martedì 7 luglio alle ore 18:30 all'evento online, organizzato da @founding, dove proveremo a der il nostro piccolo supporto alle #startup in phase di pre-seed partecipanti al programma di accelerazione. Per partecipare l'iscrizione è gratuita	tuesday july online event organize give little support startups pred phase participate acceleration program participate registration free
انا عن نفسي، اكتشفت قوتي في المشاريع التقليدية، التقليدية اقصد فيها انه ماهو مشروع ريادي جديد يحل مشكله جديدة، مافي مشروع قد سبقة فيها. وجدا ما اطيق ولا احب ادخل مشروع ريادي جديد ما فيه منافسين!	discover strength traditional traditional project mean entrepreneurial project solve problem project precede cant stand dont like enter entrepreneurial project competitors

RETRACTED

**Table 4:** Extraction of Word2Vec vector.

	Word	V1	V2
1	Renewables	0.725080668926239	1.3420028686523438
2	Industry	0.91641366481781	0.5970061421394348
3	Financialfreedom	1.4879175424575806	−1.5205949544906616
4	Solar	0.1703941971063614	0.2903654873371124
5	Socialmedia	1.018614649772644	−0.24768508970737454
6	Domainname	0.4955303072929382	−0.16176468133926392
7	Ecosystem	0.35857278108596796	0.4451853930950165
8	Solarenergy	0.14967939257621765	0.34180358052253723
9	Electricvehicles	0.2645399868488312	1.8763582706451416
10	Lifestyle	0.9395042061805724	−0.6622232794761658
11	Marketingstrategy	0.6340960860252379	−0.242161437869072
12	Forextrading	1.3747655153274536	−1.0343251228332522
13	Hardware	1.5988072156906128	1.210995316505432
14	Healthtech	0.8135859370231628	0.8424510359764099
15	Online	0.7914919257164001	−0.2414100468158722
16	Entrepreneurs	0.918533742427826	−0.08370804786682129
17	Entrepreneurship	1.011565923690796	−0.5792393088340759
19	Energy	−0.070171356201171	0.8830568194389343
20	Investors	0.7606561779975891	−0.26808339357376104
21	Forextrader	1.3127658367156982	−1.59566330909729
22	Learn	0.7077612280845642	0.5280530452728271
23	Robots	0.5793766379356384	0.9981095194816588
24	Founder	1.028773069381714	−0.0499202124774456
25	Bigdata	0.9291335344314576	0.07784397155046463
26	Renewableenergy	0.04838217794895172	0.2493981868028641
27	Blockchain	0.643086850643158	−0.5717571973800659
28	Finance	0.8881515860557556	−0.9954341053962708
32	Artificialintelligence	0.5451000928878784	0.40275973081588745
33	Healthcare	0.8982919454574585	0.10228601843118668
35	Tech	0.9358549714088441	1.6602802276611328
36	Digitalmarketing	0.9457358121871948	−0.4341220259666443
37	Investment	0.8618270754814148	−0.5015068054199219
	…	…	…

RETRACTED

**Table 5:** Experimentation with total tweets.

Num	Parameters				Word2Vec size
	Vector_size	Min_word_frequency	Window size	Epochs	
1	2	3	1	1000	3065876
2	2	5	1	1000	28278
3	2	5	1	500	28278
4	2	5	2	500	28278
5	5	5	2	500	28278
6	5	6	1	500	24814

**Table 6:** Extraction of the recommended projects.

Recommended smart city startup services	Required skills and competencies
Driverless cars	Machine learning, electrical engineering, robotics, programming
Renewble energy	Energy engineering, sustainability, green energy, chemistry, geographic information systems, technology
Health tech	Data collection, data analysis, communication, programming
Digital marketing	Social media, search engine marketing, strategy & planning, social selling, Internet

**Table 7:** Results of performance measures.

Num	Parameters				Precision	Recall	F-Measure
	Vector_size	Min frequency	Window size	Epochs			
1	2	3	1	1000	0.98	0.66	0.79
2	2	5	1	1000	0.97	0.41	0.58
3	2	5	1	500	0.97	0.41	0.58
4	2	5	2	500	0.97	0.41	0.58
5	5	5	2	500	0.97	0.41	0.58
6	5	6	1	500	0.96	0.35	0.51
Performance measures average					0.97	0.44	0.60

**Table 8:** Comparison of performance measures with existing approaches.

	Precision	Recall	F-measure
RecSPSC	0,97	0,44	0,6
CB	0,82	0,24	0,37
CF	0,87	0,19	0,31

## Data Availability

No data were used to support this study.

## References

[1] Girardi P., Temporelli A. (2017). Smartainability: a methodology for assessing the sustainability of the smart city. *Energy Procedia*.

[2] Haarstad H., Wathne M. W. (2019). Are smart city projects catalyzing urban energy sustainability?. *Energy Policy*.

[3] Hajduk S. (2020). Using multivariate statistical methods to assess the urban smartness on the example of selected European cities. *PLoS One*.

[4] Winden W. V., Buuse D. V. D. (2017). Smart city pilot projects: exploring the dimensions and conditions of scaling up. *Journal of Urban Technology*.

[5] Ahvenniemi H., Huovila A. (2020). How Do Cities Promote Urban Sustainability and Smartness? an Evaluation of the City Strategies of Six Largest Finnish Cities. *Environment, Development and Sustainability*.

[6] Yigitcanlar T. (2017). Smart cities in the making. *International Journal of Knowledge-Based Development*.

[7] Oomens I. M. F., Sadowski B. M. (2019). The importance of internal alignment in smart city initiatives: an ecosystem approach. *Telecommunications Policy*.

[8] Lytras M., Visvizi A., Sarirete A. (2019). Clustering smart city services: perceptions, expectations, responses. *Sustainability*.

RETRACTED

[9] Nicholls L., Strengers Y., Sadowski J. (2020). Social impacts and control in the smart home. *Nature Energy*.

[10] Xu Z., Gao Y., Hussain M., Cheng P. (2020). Demand side management for smart grid based on smart home appliances with renewable energy sources and an energy storage system. *Mathematical Problems in Engineering*.

[11] Li M., Tang H., Hussein A. R., Wang X. (2020). A sidechain-based decentralized authentication scheme via optimized two-way peg protocol for smart community. *IEEE Open Journal of the Communications Society*.

[12] Pereira G. V., Parycek P., Falco E., Kleinhans R. (2018). Smart governance in the context of smart cities: a literature review. *Information Polity*.

[13] Park H., Rhee S. B. (2018). IoT-based smart building environment service for occupants’ thermal comfort. *Journal of Sensors*.

[14] Kusiak A. (2018). Smart manufacturing. *International Journal of Production Research*.

[15] Taylor M. (2018). Climate-smart agriculture: what is it good for?. *Journal of Peasant Studies*.

[16] Sharma N., Kaushik I., Bhushan B., Gautam S., Khamparia A. (2020). Applicability of WSN and biometric models in the field of healthcare. *Deep Learning Strategies for Security Enhancement in Wireless Sensor Networks*.

[17] Khamparia A., Singh P. K., Rani P., Samanta D., Khanna A., Bhushan B. (2020). An internet of health things‐driven deep learning framework for detection and classification of skin cancer using transfer learning”. *Transactions on Emerging Telecommunications Technologies*.

[18] Goyal S., Sharma N., Bhushan B., Shankar A., Sagayam M. (2021). Iot enabled technology in secured healthcare: applications, challenges and future directions. *Cognitive Internet of Medical Things for Smart Healthcare*.

[19] Kumar A., Krishnamurthi R., Nayyar A., Sharma K., Grover V., Hossain E. (2020). A novel smart healthcare design, simulation, and implementation using healthcare 4.0 processes. *IEEE Access*.

[20] Tian S., Yang W., Micheal J. (2019). Smart healthcare: making medical care more intelligent. *Global Health Journal*.

[21] Islam M. M., Rahaman A., Islam M. R. (2020). Development of smart healthcare monitoring system in IoT environment. *SN computer science*.

[22] Alanazi S. A., Kamruzzaman M. M., Alruwaili M., Alshammari N., Alqahtani S. A., Karime A. (2020). Measuring and preventing COVID-19 using the SIR model and machine learning in smart health care. *Journal of healthcare engineering*.

[23] Du X., Chen B., Ma M., Zhang Y. (2021). Research on the application of blockchain in smart healthcare: constructing a hierarchical framework. *Journal of Healthcare Engineering*.

[24] Yuan Y., Lu Y., Chow T. E., Ye C., Alyaqout A., Liu Y. (2020). The missing parts from social media-enabled smart cities: who, where, when, and what?. *Annals of the Association of American Geographers*.

RETRACTED

[25] Chifor B., Bica I., Patriciu V. (2017). Sensing service architecture for smart cities using social network platforms. *Soft Computing*.

[26] Smailhodzic E., Hooijsma W., Boonstra A., Langley D. J. (2016). Social media use in healthcare: a systematic review of effects on patients and on their relationship with healthcare professionals. *BMC Health Services Research*.

[27] Lin X., Kishore R. (2021). Social media-enabled healthcare: a conceptual model of social media affordances, online social support, and health behaviors and outcomes. *Technological Forecasting and Social Change*.

[28] Gupta A., Katarya R. (2020). Social media based surveillance systems for healthcare using machine learning: a systematic review. *Journal of Biomedical Informatics*.

[29] Chen X., Lun Y., Yan J., Hao T., Weng H. (2019). Discovering thematic change and evolution of utilizing social media for healthcare research. *BMC Medical Informatics and Decision Making*.

[30] Pershad Y., Hangge P., Albadawi H., Oklu R. (2018). Social medicine: twitter in healthcare. *Journal of Clinical Medicine*.

[31] Molinillo S., Sánchez R. A., Morrison A. M., Stefaniak J. A. C. (2019). Smart city communication via social media: analysing residents’ and visitors’ engagement. *Cities*.

[32] Pujol F. A., Mora H., Pertegal M. L. (2019). A soft computing approach to violence detection in social media for smart cities. *Soft Computing*.

[33] Wang D., Al-Rubaie A., Clarke S. S., Davies J. (2017). Real-time traffic event detection from social media. *ACM Transactions on Internet Technology*.

[34] Jain S., Sinha A. (2019). Social network sustainability for transport planning with complex interconnections. *Sustainable Computing: Informatics and Systems*.

[35] Stojanovski D., Strezoski G., Madjarov G., Dimitrovski I. (2018). Emotion identification in twitter messages for smart city applications. *Information Innovation Technology in Smart Cities*.

[36] Alkhatib M., Barachi M. E., Shaalan K. (2019). An Arabic social media based framework for incidents and events monitoring in smart cities. *Journal of Cleaner Production*.

[37] Costa D. D. (2018). Twittersensing: an event-based approach for wireless sensor networks optimization exploiting social media in smart city applications. *Sensors*.

[38] Lytras M. D. P. (2018). Social networks research for sustainable smart education. *Sustainability*.

[39] Visvizi A., Jussila J., Lytras M. D., Ijäs M. (2020). Tweeting and mining OECD-related microcontent in the post-truth era: a cloud-based app. *Computers in Human Behavior*.

RETRACTED

[40] SDB (2021). The social development bank. https://www.sdb.gov.sa/en-us/our-products/projects/productive-loans.

[41] (2021). Almaal.org. Small business support. https://www.almaal.org/support-small-businesses-in-saudi-arabia.

[42] Mohamed M. H., H Khafagy M., Ibrahim M. H. Recommender systems challenges and solutions survey.

[43] Tarus J. K., Niu Z., Mustafa G. (2018). Knowledge-based recommendation: a review of ontology-based recommender systems for e-learning. *Artificial Intelligence Review*.

[44] Aggarwal C. C. (2016). Recommender systems. *Champion: Springer International Publishing*.

[45] Yang X., Guo Y., Liu Y., Steck H. (2014). A survey of collaborative filtering based social recommender systems. *Computer Communications*.

[46] Javed U., Shaukat K., Hameed I. (2021). A review of content-based and context-based recommendation systems. *International Journal of Emerging Technologies in Learning (iJET)*.

[47] Kim H. J., Kim T. S., Sohn S. Y. (2020). Recommendation of startups as technology cooperation candidates from the perspectives of similarity and potential: a deep learning approach. *Decision Support Systems*.

[48] Wu S., Li H., Liu L. (2020). A venture capital recommendation algorithm based on heterogeneous information network. *International Journal of Computers, Communications & Control*.

[49] Xu S., Zhang Q., Liü L., Lü M. S. (2020). Recommending investors for new startups by integrating network diffusion and investors’ domain preference. *Information Sciences*.

[50] Zhong H., Liu C., Zhong J., Xiong H. (2018). Which startup to invest in: a personalized portfolio strategy. *Annals of Operations Research*.

[51] Lasmar E. L., Paula F. O. D., Rosa R. L., Abrahão J. I., Rodríguez D. Z. (2019). RsRS: ridesharing recommendation system based on social networks to improve the user’s QoE. *IEEE Transactions on Intelligent Transportation Systems*.

[52] Zhao X., Ma Z., Zhang Z. (2018). A novel recommendation system in location-based social networks using distributed ELM. *Memetic computing*.

[53] Ke G., Du H., Chen Y. (2021). Cross-platform dynamic goods recommendation system based on reinforcement learning and social networks. *Applied Soft Computing*.

[54] Statista.com. https://www.statista.com/topics/737/twitter/Visitedmarch2021.

[55] Omnicoreagency.com. https://www.omnicoreagency.com/twitter-statistics/Visitedmarch2021.

[56] Vijayarani S., Janani R. (2016). Text mining: open source tokenization tools-an analysis. *Advanced Computational Intelligence: International Journal*.

[57] Akhmetov I., Pak A., Ualiyeva I. (2020). Highly language-independent word lemmatization using a machine-learning classifier. *Computación y Sistemas*.

RETRACTED

[58] Celano G. G. A gradient boosting-seq2seq system for latin pos tagging and lemmatization.

[59] Church K. W. (2017). Word2Vec. *Natural Language Engineering*.

[60] Ayyadevara V. K. (2018). Word2vec, pro machine learning algorithms. *Pro Machine Learning Algorithms*.

[61] Chang C. Y., Lee S. J., Lai C. C. Weighted word2vec based on the distance of words.

[62] Zuo X., Zhang S., Xia J. (2017). The enhancement of TextRank algorithm by using word2vec and its application on topic extraction. *Journal of Physics: Conference Series*.

[63] Suleiman D., Awajan A. A. Using part of speech tagging for improving Word2vec model.

[64] Fipa (2000). *FIPA Nomadic Application Support Specification*.

[65] OWL-Time (2006). *Time Ontology in OWL*.

[66] Haller A., Janowicz K., Cox S. J. (2019). The modular SSN ontology: a joint W3C and OGC standard specifying the semantics of sensors, observations, sampling, and actuation. *Semantic Web*.

[67] Kolozali S., Bermudez M. E, Puschmann D., Ganz F., Barnaghi P. A knowledge-based approach for real-time iot data stream annotation and processing.

[68] Millstein F. (2020). *Natural Language Processing with python: Natural Language Processing Using NLTK*.

